The article "Silencing the ADAM9 Gene through CRISPR/Cas9 Protects Mice from Alcohol-Induced Acute Liver Injury" was published in 2022. Journal: Biomed Res Int.

# Silencing the ADAM9 Gene through CRISPR/Cas9 Protects Mice from Alcohol-Induced Acute Liver Injury

**DOI:** 10.1155/2022/5110161

**Published:** 2022-06-06

**Authors:** Yong-Yong Zhang, San-Qiang Li, Ying Song, Ping Wang, Xiao-Gai Song, Wen-Feng Zhu, Dong-Mei Wang

**Affiliations:** ^1^The Molecular Medicine Key Laboratory of Liver Injury and Repair, School of Basic Medical Sciences, Henan University of Science and Technology, Luoyang 471003, China; ^2^Orthopedic Institute of Henan Province, Luoyang, 471003 Henan, China; ^3^Henan Center for Engineering and Technology Research on Prevention and Treatment of Liver Diseases, Luoyang 471003, China

## Abstract

Alcoholic liver injury is a major global public health concern at present. The ADAM9 gene plays a crucial role in the occurrence and development of various liver diseases, but its role in acute alcoholic liver injury remains ambiguous. In this study, a chimeric single-guide RNA targeting the genomic regions of mouse ADAM9 was designed using the clustered regularly interspaced short palindromic repeats (CRISPR)/CRISPR-associated protein 9 (Cas9) technology. Next, the role of ADAM9 in acute alcoholic liver injury *in vitro* in cultured mouse cells and *in vivo* in a hydrodynamic injection-based alcoholic liver injury mouse model was documented. The findings of this study suggest that ADAM9 induces by regulating cell proliferation, apoptosis, and stress metabolism in mice. Thus, inhibiting the expression of ADAM9 gene using CRISPR/Cas9 can attenuate alcohol-induced acute liver injury in mice.

## 1. Introduction

Alcoholic liver disease (ALD) has high rates of morbidity and mortality and has become a severe and challenging health problem worldwide [1]. In western countries, 50%–75% cases of cirrhosis arise because of excessive alcohol consumption, and approximately 15,000–20,000 Americans die annually of ALD. In China, following viral hepatitis, ALD is the second leading cause of liver injury. ALD refers to a series of liver damage caused by long-term or excessive drinking, including hepatic steatosis, steatohepatitis, and fibrosis, which could advance to hepatocellular carcinoma in severe cases [2–4]. Several studies have investigated the mechanism of alcoholic liver injury and have shown that it is closely associated with oxidative stress, apoptosis and proliferation, production of a large amount of reactive oxygen species, and alcohol metabolites [5]. However, the pathogenesis of liver injury remains unclear. ADAM9, a highly studied a disintegrin and metalloproteinase (ADAM) family member, is involved in the development and molecular mechanisms of various diseases [6]. Previously, ADAM9 was found to regulate hepatocyte proliferation and apoptosis, angiogenesis, and cytochrome P450 family 2 subfamily E member 1 (CYP2E1) expression by activating the interleukin-6 (IL-6) transduction signal and played an important protective role in CCl4-induced acute liver injury in mice [7]. Because ALD is similar to CCL4-induced chemical liver injury, this study was conducted to further explore the role of ADAM9 in the process of alcohol-induced liver injury.

The article "Silencing the ADAM9 Gene through CRISPR/Cas9 Protects Mice from Alcohol-Induced Acute Liver Injury" was published in 2022. Journal: Biomed Res Int.

The ADAM family members, also known as metalloprotease-like disintegrin-like cysteine-rich proteins, are type I transmembrane secretory glycoproteins that possess integrin and metalloproteinase functions. The proteins encoded by the ADAM gene usually contain 800–1200 amino acids and sequentially conserved domains [8] named, from the *N*-terminus to the *C*-terminus, as follows: signal domain, prodomain, metalloproteinase domain, disintegrin domain, cysteine-rich domain, epidermal growth factor-like domain, transmembrane domain, and cytoplasmic tail [9]. ADAM proteins are widely expressed in various tissues and play several different roles. They are extensively involved in the inflammatory response, allergies, tumor development and metastasis, and immune diseases [10]. Studies have found that ADAM9 is associated with the occurrence, development, and metastasis of hepatocellular carcinoma [11, 12] and that many liver cancers often develop gradually from ALD [13]. Therefore, the function of ADAM9 during liver injury was studied. Understanding its molecular mechanisms could allow us to detail the liver injury process and provide a theoretical basis to prevent its further development into liver cancer.

## 2. Materials and Methods

### 2.1. Cell Culture and Transfection

Cell culture: mouse C2C12 myoblasts were purified at the Shanghai Fudan University Biomedical Research Institute and maintained in Dulbecco's modified Eagle medium (DMEM) supplemented with 10% fetal bovine serum and 100 IU/mL penicillin (Solarbio, Shanghai, China). Cells were incubated at 5% CO_2_ and saturated humidity at 37°C with 100 *μ*g/mL streptomycin. Transfection was performed using Lipofectamine 3000 (Thermo Fisher Scientific, USA).

### 2.2. Single-Guide RNA (sgRNA) Design and Plasmid Construction

To design the sgRNAs targeting the ADAM9 gene sequences (obtained from NCBI), the online tool developed by Prof. Feng Zhang (http://crispr.mit.edu/) was used. To disrupt the *Pep_M12B*_propep and *ZnMc* domains, the gene on exon 2 and exon 12 (corresponding to residues 44 and 406) needed to be cleaved. Following a comparative analysis, three clustered regularly interspaced short palindromic repeat (CRISPR) sequences were synthesized (Figure 1). In total, three sgRNAs were designed and three 3-in-1 plasmids were synthesized: pYSY-CMV-Cas9-U6-Adam9-sgRNA1-EFla-Puromycin, pYSY-CMV-Cas9-U6-Adam9-sgRNA2-EFla-Puromycin, and pYSY-CMV-Cas9-U6-Adam9-sgRNA3-EFla-Puromycin, where CMV, U6, and EFla were the Cas9, Adam9-sgRNA1, and puromycin gene promoters, respectively. The synthesized plasmids were amplified by polymerase chain reaction (PCR) and verified by electrophoresis. Positive clones were found at approximately 100 bp (Figure 2).

The article "Silencing the ADAM9 Gene through CRISPR/Cas9 Protects Mice from Alcohol-Induced Acute Liver Injury" was published in 2022. Journal: Biomed Res Int.

### 2.3. Effective Plasmid Screening

Equal proportions of the three plasmids were mixed and transfected into mouse C2C12 myoblasts using Lipofectamine 3000. When the concentration of transfected cells reached a confluency of approximately 70%, they were treated with puromycin (50 *μ*g/*μ*L) to screen for single-cell cloning. After extensive cell expansion, cellular genomic DNA was extracted using a genomic DNA extraction kit (Aisijin Biotech Ltd., Shenzhen, China) and PCR was performed. The following primer sequences were used: ADAM9-Exon2-Forward: 5′-TGACCTGGAACTCACAAA-3′, ADAM9-Exon2-Reverse: 5′-TCCACTCCCTTCATTCTG-3′, ADAM9-Exon11-Forward: 5′-GGTCTGTTGATGCCTGAT-3′, ADAM9-Exon11-Reverse 5′-ATGTAATATGCCCTACCC-3′. PCR was performed in 25 *μ*L of a solution containing 1 *μ*L Oligo-F, 1 *μ*L Oligo-R, 1 *μ*L cDNA, 12.5 *μ*L 2× Es Taq MasterMix, and 9.5 *μ*L RNase-free H_2_O (all from Shanghai Shenggong Biotech Ltd.), under the following conditions: 30 cycles at 94°C for 30 s, 52.5°C for 30 s, and 70°C for 30 s, followed by a 10 min extension step at 70°C. After agarose gel electrophoresis, the PCR products were recovered using a gel extraction kit (OMEGA, USA) and sent to Shanghai Shenggong Biotech Ltd. for sequencing.

Finally, only the sgRNA3 sequence was found to differ significantly from the original sequence (Figure 3). The C2C12 cells were transfected with the sgRNA3 plasmid again to confirm its efficiency and the proteins extracted from stably expressing cells for the purpose of immunoblotting. The sgRNA3-transfected cells had considerably lower levels of ADAM9 than normal cells (Figure 4).

### 2.4. Animals and Experimental Design

Male BALB/c mice (6–8 weeks old, 22 ± 2 g) were purchased from the experimental animal center of the Henan province. All animals were allowed to feed on laboratory chow and allowed 1 week to adapt to the environment before the experiments. All the protocols complied with the guidelines of the National Animal Care and Use Committee of China. In addition, all the animals received care in compliance with the Principles of Laboratory Animal Care.

The mice were randomly divided into three groups (10 mice/group): normal group (no treatment), saline+alcohol group (positive control group subjected to a tail vein injection of normal saline and alcoholic gavage), and ADAM9-sgRNA3+alcohol group (experimental group subjected to a tail vein injection of 60 ng/mice of sgRNA3 plasmids followed by alcoholic gavage) [14]. In the positive control and experimental groups, the mice were fed with 56% (*v*/*v*) alcohol (Red Star Erguotou Liquor, 56°C, Beijing, China) (24 ml/kg) via oral gavage at the end of the third day after the tail vein injection. The mice were starved for 24 h after alcohol gavage and euthanized by cervical dislocation to collect blood and harvest liver tissues.

The article "Silencing the ADAM9 Gene through CRISPR/Cas9 Protects Mice from Alcohol-Induced Acute Liver Injury" was published in 2022. Journal: Biomed Res Int.

### 2.5. Serum Transaminase Activity Detection

Blood samples were collected from the eyeballs of all the mice at 24 h after alcohol administration, and the completely coagulated blood (4000 rpm, 5 min) was centrifuged to obtain serum. The serum aspartate aminotransferase (AST) and alanine aminotransferase (ALT) activities were determined using a commercial assay kit (Xinyu Biological Technology Ltd., Shanghai, China) [15]. This kit is based on double antibody sandwich enzyme-linked immunosorbent assay method. The anti-mouse ALT antibody is coated on the micro enzyme-labeled plate to capture ALT from the serum sample. Then, the biotinylated anti-mouse ALT antibody followed by horseradish peroxidase-labeled avidin was added. Biotin specifically interacts with avidin to form an immune complex, and finally, the chromogenic substrate was added. The optical density (OD) was measured at 450 nm using a microplate reader, and ALT concentration in mice was proportional to the OD. The enzyme activity was expressed in international unit per liter (IU/L).

### 2.6. Histopathological Examination

The isolated mouse liver samples were fixed in 10% formaldehyde for 24 h and dehydrated, and tissue wax blocks were then prepared. Sections of 5 *μ*m thickness were cut from each paraffin-embedded tissue and stained with hematoxylin and eosin [16, 17]. Hepatocyte necrosis was photographed using a digital microscope system (Moticam Pro Motic, Xiamen, China), and the hepatocyte necrosis rate was scored using the following scale: no lesion = 0, <2 lesions/visual field = 1, 2–4 lesions/visual field = 2, and >4 lesions/visual field = 3.

### 2.7. Hoechst 33258 Staining Assay for Hepatocyte Apoptosis

Apoptosis in the hepatocytes of the different groups of mice was analyzed using a commercial kit (BEYOTIME, Shanghai, China) [18]. The stained sections were assessed microscopically, and photographs were taken using a digital image capture system (Olympus). A microscope was used for counting normal and apoptotic cells. The apoptotic rate was calculated as follows: apoptotic rate = [number of apoptotic cells/total number of cells] × 100%. This experiment was repeated thrice.

The article "Silencing the ADAM9 Gene through CRISPR/Cas9 Protects Mice from Alcohol-Induced Acute Liver Injury" was published in 2022. Journal: Biomed Res Int.

### 2.8. Periodic Acid–Schiff (PAS) Staining

After conventional gradient dewaxing and hydration, the tissue sections were incubated in 0.8% periodic acid for 15 min, then stained with Schiff reagent for 20 min, and finally counterstained with hematoxylin [19]. Using an optical microscope, 10 representative fields of each group were randomly selected for observation, and their optical density was analyzed using the Motic Images Advanced 3.2 software (Moticam Pro Motic, Xiamen, China). This experiment was repeated three times.

### 2.9. Western Blotting

Proteins were quantified using a BCA Protein Assay Kit (Solarbio, Shanghai, China), and 50 *μ*g of the sample was subjected to sodium dodecyl sulfate-polyacrylamide gel electrophoresis; the proteins were then electrotransferred onto a nitrocellulose membrane. Next, the membrane was treated with monoclonal antibodies against mouse ADAM9, heat shock protein 27 (HSP27), heat shock protein 70 (HSP70), proliferating cell nuclear antigen (PCNA), B cell lymphoma protein 2 (Bcl-2), Bcl-2-associated X (Bax), caspase-3, vascular endothelial growth factor (VEGF), and phosphorylated signal transducer and activator of transcription 3 (p-STAT3) (Santa Cruz). The signal was detected by employing a horseradish peroxidase detection system using diaminobenzidine (Sigma). The protein bands were quantified with the Gel-Pro Analyzer software 4.0 (Media Cybernetics Inc., Bethesda, MD) and their intensities normalized to beta-actin. Every experiment was repeated thrice [7].

### 2.10. In Vitro Experiments

The L02 hepatocytes obtained from Shanghai Fudan University Biomedical Research Institute were purified and cultured under 5% CO_2_ at 37°C in modified DMEM supplemented with 15% fetal bovine serum, 100 units/mL penicillin, and 100 units/mL streptomycin. When the cells on the 10 cm^2^ dish reached a confluency of 70%, they were separated into four groups: normal (nontransfected, untreated), normal+ADAM9-sgRNA3 (plasmid-transfected, untreated), saline+alcohol (nontransfected, alcohol-treated), and ADAM9-sgRNA+alcohol (plasmid-transfected, alcohol-treated) groups. The L02 hepatocytes were transfected with the screened sgRNA3 plasmid (plasmid-transfected cells), and the monoclonal cell line deficient in ADAM9 gene was screened and cultured using the aforementioned monoclonal cell screening method. When cells reached 70% confluency, they were treated with alcohol (30 *μ*L/mL) for 24 h (alcohol-treated cells).

### 2.11. Statistical Analysis

All the data were expressed as the mean ± SEM. Comparisons between two groups were conducted using the independent sample *t*-test, and the one-way analysis of variance (ANOVA) test was used for comparisons between more than two groups. *P* values of <0.05 and <0.01 were considered statistically significant and highly significant, respectively. All statistical calculations were performed using the SPSS 19.0 software (SPSS, Inc., Chicago, IL, USA).

The article "Silencing the ADAM9 Gene through CRISPR/Cas9 Protects Mice from Alcohol-Induced Acute Liver Injury" was published in 2022. Journal: Biomed Res Int.

## 3. Results

### 3.1. Serum ALT and AST Enzyme Activities in Mice

Figure 5 shows that the positive control and experimental groups (both of which received ethanol treatment) had significantly higher serum AST and ALT levels than the normal group (*P* < 0.05 and *P* < 0.01). Moreover, the experimental group had significantly lower serum AST and ALT levels than the positive control group (*P* < 0.01).

### 3.2. HE Staining for the Detection of Hepatocyte Necrosis Rate

Figure 6 shows that the positive control and experimental groups showed the presence of liver injuries that the normal group did not (*P* < 0.05 or *P* < 0.01). Besides, the experimental group had a significantly lower hepatocyte necrosis score than the positive control group (*P* < 0.01).

### 3.3. PAS Staining for Hepatic Glycogen Detection

The experimental and positive control groups showed significantly higher hepatic glycogen consumption than the negative control group (*P* < 0.05 and *P* < 0.01; Figure 7). However, hepatic glycogen consumption was lower in the experimental group than in the positive control group (*P* < 0.05; Figure 7).

### 3.4. Hoechst 33258 Staining for Hepatocyte Apoptosis Detection

Figure 8 shows that ethanol treatment markedly increased the hepatocyte apoptosis rate (experimental and positive control groups *vs.* negative control group: *P* < 0.05 and *P* < 0.01, respectively). However, the hepatocyte apoptosis rate was lower in the experimental group than in the positive control group (*P* < 0.05).

### 3.5. Western Blotting Results of the Experiment on Mice

Figure 9 shows that ADAM9 expression was higher in the positive control and experimental groups than in the negative control group (*P* < 0.05 and *P* < 0.01). Besides, ADAM9 expression was significantly lower in the experimental group than in the positive control group (*P* < 0.05). Thus, injecting the plasmid into the tail vein was found to considerably inhibit the expression of ADAM9 gene in the mouse liver tissue. Meanwhile, the positive control and experimental groups had significantly higher expression levels of HSP27, HSP70, Bax, caspase-3, and p-STAT3 than the negative control group and lower expression levels of PCNA, Bcl-2, and VEGF. In addition, the experimental group had higher expression levels of HSP27, HSP70, PCNA, Bcl-2, VEGF, and p-STAT3 than the positive control group and lower expression levels of Bax and caspase-3 (Figure 9).

The article "Silencing the ADAM9 Gene through CRISPR/Cas9 Protects Mice from Alcohol-Induced Acute Liver Injury" was published in 2022. Journal: Biomed Res Int.

### 3.6. Western Blotting Results of L02 Hepatocytes

Figure 10 shows a significant increase in the expression of ADAM9 in alcohol-treated stem L02 cells, whereas the expression of the ADAM9 protein was significantly inhibited when the cells were transfected with sgRNA3 plasmid (*P* < 0.05 and *P* < 0.01). The positive control group had significantly higher expression levels of HSP27, HSP70, Bax, caspase-3, and p-STAT3 and lower expression levels of PCNA, Bcl-2, and VEGF than the negative control group (*P* < 0.05 and *P* < 0.01). In the experimental group, the expression levels of HSP27, HSP70, Bax, caspase-3, and p-STAT3 were significantly increased, whereas the expression levels of PCNA, Bcl-2, and VEGF were decreased (*P* < 0.05 and *P* < 0.01), which is similar to that observed in the positive CRISPR control group. When the two groups in which ADAM9 gene knockout was performed were compared with the two groups with the ADAM9 gene, i.e., when the normal+sgRNA3 group was compared with the negative control group and the experimental group was compared with the positive control group, the expressions of the HSP27, HSP70, PCNA, Bcl-2, VEGF, and p-STAT3 proteins were significantly increased, whereas only the expressions of Bax and caspase-3 were significantly decreased (*P* < 0.05 and *P* < 0.01).

## 4. Discussion

CRISPR/Cas9 is a recently developed genome editing technology that uses sgRNA and the Cas9 nuclease for identifying and editing specific DNA sites; it provides a novel platform for human gene editing. However, because it frequently affects off-target DNA, three sgRNAs were designed and the most successful sgRNA was selected [20, 21] (Figures 1 and 2). sgRNA3 successfully inhibited the expression of ADAM9 gene in the mouse liver (Figure 3). Mouse C2C12 cells were transfected with the three successfully constructed plasmids, screened using puromycin, and the cell DNA extracted for sequencing after the formation of a stable clone. On comparing this sequence with the original sequence, the sgRNA3 plasmid was found to knock out the ADAM9 gene (Figure 3). Next, the cellular protein was extracted and the validity of the sgRNA3 plasmid was verified again at the protein level (Figures 4, 9(a), 9(b), 10(a), and 10(b)).

The effect of the inhibition of ADAM9 gene expression was initially observed on alcohol-induced acute liver injury. AST and ALT are both tissue enzymes that catalyze the exchange of amino and keto groups between alpha amino and keto acids. Tissue toxicity causes the release of these enzymes into the general circulation, thereby increasing the levels of these enzymes [22]. The results showed that the experimental group had significantly lower serum AST and ALT levels (*P* < 0.05, Figure 5) and hepatocyte necrosis score (*P* < 0.05, Figure 6) than the positive control group. However, the liver glycogen level in the experimental group was significantly higher than that in the positive control group. Glycogen synthesis in the liver is the main form of energy storage in animals. Liver glycogen content decreased proportionally with increase in the severity of alcoholic liver disease in the early stage [23, 24]. The results of this study showed that alcohol-induced injury decreased the hepatic glycogen content in mice; however, the inhibition of ADAM9 gene expression partially prevented this decrease. These results indicate that ADAM9-sgRNA3 significantly attenuated the severity of alcohol-induced liver injury and suggest that ADAM9 contributes to alcohol-induced liver injury promotion.

The article "Silencing the ADAM9 Gene through CRISPR/Cas9 Protects Mice from Alcohol-Induced Acute Liver Injury" was published in 2022. Journal: Biomed Res Int.

The findings of this study showed that after inhibiting the expression of the ADAM9 gene in alcohol-induced acute liver injury, the expression of HSP27 and HSP70 further increased in comparison with the positive control group (*P* < 0.05 and *P* < 0.01) (Figures 9(a), 9(c), 9(d), 10(a), 10(c), and 10(d)). HSP27 and HSP70 are molecular chaperones that are essential for accurate three-dimensional folding of nascent polypeptide chains and proteins and the repair process after protein damage [25]. These molecular chaperones protect proteins and maintain normal cellular physiological activity when external factors promote their mass production. The results of this study showed that silencing the ADAM9 gene increased the expression of HSP27 and HSP70 in the liver of mice. Therefore, ADAM9 may promote liver damage during acute alcoholic liver injury by reducing the expression of heat shock proteins.

The results of this study showed that silencing ADAM9 significantly reduced the apoptosis rate (experimental group *vs*. positive control group, *P* < 0.05) (Figure 8). Casp3, Bax, and Bcl-2 are important factors associated with apoptosis. Inhibition of the expression of the ADAM9 gene was shown to significantly reduce the Bax and caspase-3 expression levels and increase those of Bcl-2 (*P* < 0.05 and *P* < 0.01) (Figures 9(a), 9(f), 9(g), 9(h), 10(a), 10(f), 10(g), and 10(h)). Caspase-3 is a member of the interleukin-1 beta-converting enzyme or cell death effector-3 family, which plays an irreplaceable role in apoptosis, and caspase-3 is the most important terminal cleavage enzyme in the process of apoptosis [26]. Insect Sf9 cells were transfected with caspase-3 gene to induce apoptosis, and this process could be blocked by Bcl-2. Bax and Bcl-2 are important proapoptotic and antiapoptotic markers, respectively, which contribute significantly to the regulation of apoptosis [27, 28]. Therefore, inhibiting the expression of the ADAM9 gene can inhibit apoptosis by upregulating antiapoptotic inhibitors and downregulating proapoptotic factors.

The article "Silencing the ADAM9 Gene through CRISPR/Cas9 Protects Mice from Alcohol-Induced Acute Liver Injury" was published in 2022. Journal: Biomed Res Int.

The results of this study showed that ADAM9 knockout significantly upregulated the expression of PCNA in alcohol-induced acute liver injury in mice (*P* < 0.05 and *P* < 0.01) (Figures 9(a), 9(e), 10(a), and 10(e)). PCNA, synthesized in the nucleus of mammalian cells, plays a crucial role in the cell proliferation cycle. Its expression levels are lower in the G2 to M phase and peak in the S phase, making it a good indicator of the proliferative capacity of cells [29]. It was further demonstrated that the knockout of the ADAM9 gene could promote hepatocyte proliferation in alcohol-induced acute liver injury; i.e., the knockout of the ADAM9 gene can alleviate alcohol-induced acute liver injury.

The findings of this study also showed that inhibition of the ADAM9 gene can significantly promote the expression of VEGF in alcohol-induced acute liver injury (*P* < 0.05 and *P* < 0.01) (Figures 9(a), 9(i), 10(a), and 10(i)). VEGF is a major cytokine that has multiple functions such as promoting neovascularization, increasing vascular permeability, promoting endothelial cell proliferation, and inhibiting apoptosis. In patients with chronic hepatitis, the expression of VEGF is more pronounced in hepatocytes and sinus spaces in hepatic vascular inflammation, destruction, and obstruction, and its expression in liver tissue increases with the aggravation of liver tissue degeneration and necrosis [30]. The findings of this study suggested that inhibiting the expression of ADAM9 gene significantly increased the expression of VEGF (experimental group vs. positive control group, *P* < 0.05), indicating that ADAM9 promotes liver injury by inhibiting the expression of VEGF during alcoholic liver injury.

The experimental group had significantly higher phosphorylated signal transducer and activator of transcription 3 (p-STAT-3) protein expression levels than the positive control group in alcohol-induced acute liver injury (*P* < 0.05 and *P* < 0.01) (Figures 9(a), 9(j), 10(a), and 10(j)). p-STAT-3 is a hallmark of the IL-6 signaling pathway activation. Alcohol-stimulated hepatocytes produce multiple factors that activate the IL-6 pathway, including p-STAT3. In the nucleus, activated STAT stimulates the expression of various genes, effectively alleviating inflammatory and cellular damage during alcoholic liver injury [31]. Thus, inhibiting the expression of ADAM9 enhanced the activation of the IL-6 signaling pathway during acute alcoholic liver injury. Therefore, ADAM9 promotes liver injury by reducing the activation of the IL-6 signaling pathway during acute alcoholic liver injury.

The article "Silencing the ADAM9 Gene through CRISPR/Cas9 Protects Mice from Alcohol-Induced Acute Liver Injury" was published in 2022. Journal: Biomed Res Int.

## 5. Conclusion

This study is the first to elucidate the role of ADAM9 in acute alcoholic liver injury and its related molecular mechanisms. ADAM9 promotes liver damage by regulating the expression of genes associated with cell proliferation, apoptosis, stress, and metabolism during acute alcoholic liver injury in mice. Inhibiting the expression of ADAM9 gene using CRISPR/Cas9 technology successfully attenuated alcohol-induced acute liver injury in mice.

## Figures and Tables

**Figure 1:** CRISPR sequences of the mouse ADAM9 gene. The underlined portion and yellow highlights indicate the CRISPR sequences, and the red highlight indicates the protospacer adjacent motif (PAM) sequence GG (RC: CCN).

**Figure 2:** Electrophoresis profiles of transformant positive clones obtained by PCR. The band of approximately 100 bp was a positive clone, and the leftmost lane contained the DNA marker: 100, 250, 500, 750, 1000, 1500, 2000, 3000, and 5000 bp. Lanes 2–6: pYSY-CMV-Cas9-U6-ADAM9-gRNA1-EFla-Puromycin clones; lanes 7–11: pYSY-CMV-Cas9-U6-ADAM9-gRNA2-EFla-Puromycin clones; lanes 12–15: pYSY-CMV-Cas9-U6-ADAM9-gRNA3-EFla-Puromycin clones.

**Figure 3:** ADAM9 DNA sequence alignment results. Wild type: the ADAM9 DNA sequence of wild mice. sgRNA inhibition: ADAM9 DNA sequence of mouse C2C12 myoblast transfected with sgRNA 3. Sequencing results compared using the DNAssist software.

**Figure 4:** ADAM9 protein expression in mouse C2C12 myoblasts transfected with ADAM9-sgRNA3. (a) Detection of ADAM9 protein expression in normal C2C12 cells and C2C12 cells transfected with sgRNA3 by western blotting. (b) ADAM9 expression levels were quantified using Gel-Pro Analyzer 4.0 software (Media Cybernetics Inc.). Band intensities were normalized to *β*-actin. AU = arbitrary unit. ^∗∗^*P* < 0.01: significant differences between normal C2C12 cells and C2C12 cells transfected with sgRNA3.

**Figure 5:** Serum (a) AST and (b) ALT levels in the mice 24 h after alcohol treatment. ^∗∗^*P* < 0.01 and ^∗^*P* < 0.05: significant differences between the positive control or experimental group and the negative control group. ^##^*P* < 0.01: significant difference between the experimental and positive control groups. Every experiment was repeated three times.

**Figure 6:** Histologic examination of liver injuries in the mice 24 h after alcohol treatment. HE staining in the (a) negative control group, (b) positive control group, and (c) experimental group. (d) Necrotic score. ^∗∗^*P* < 0.01 and ^∗^*P* < 0.05: significant differences between the positive control or experimental group and the negative control group. ^##^*P* < 0.01: significant difference between the experimental and positive control groups. Every experiment was repeated three times (scale bar: 50 *μ*m).

The article "Silencing the ADAM9 Gene through CRISPR/Cas9 Protects Mice from Alcohol-Induced Acute Liver Injury" was published in 2022. Journal: Biomed Res Int.

**Figure 7:** Glycogen quantification in liver sections prepared from mice 24 h after alcohol treatment. PAS staining in the (a) negative control group, (b) positive control group, and (c) experimental group. (d) Staining quantification using the Motic Images Advanced 3.2 software (Motic China Group Co., Ltd., Xiamen, China). ^∗∗^*P* < 0.01 and ^∗^*P* < 0.05: significant differences between the positive control or experimental group and the negative control group. ^#^*P* < 0.01: significant difference between the experimental and positive control groups. Every experiment was repeated three times (scale bar: 50 *μ*m).

**Figure 8:** Apoptosis analysis of liver sections from mice 24 h after alcohol treatment. Hoechst 33258 staining in the (a) negative control group, (b) positive control group, and (c) experimental group. (d) Apoptotic rate. ^∗∗^*P* < 0.01 and ^∗^*P* < 0.05: significant differences between the positive control or experimental group and the negative control group. ^#^*P* < 0.01: significant difference between the experimental and positive control groups. Every experiment was repeated three times (scale bar: 50 *μ*m).

**Figure 9:** The influence of alcohol on the expression of ADAM9, HSP27, HSP70, PCNA, Bax, Bcl-2, caspase-3, VEGF, and p-STAT3 in the liver of mice 24 h after alcohol treatment. (a) Western blotting results. The expression levels of (b) ADAM9, (c) HSP27, (d) HSP70, (e) PCNA, (f) Bax, (g) Bcl-2, (h) caspase-3, (i) VEGF, and (j) p-STAT3 quantified with the Gel-Pro Analyzer 4.0 software (Media Cybernetics Inc.). Band intensities normalized to *β*-actin. AU = arbitrary unit. ^∗∗^*P* < 0.01 and ^∗^*P* < 0.05: significant differences between the positive control or experimental group and the negative control group. ^##^*P* < 0.01 and ^#^*P* < 0.05: significant differences between the experimental and positive control groups.

**Figure 10:** In vitro analysis of the effects of alcohol on the expression levels of ADAM9, HSP27, HSP70, PCNA, Bax, Bcl-2, caspase-3, VEGF, and p-STAT3 in hepatic L02 cells. (a) Western blotting results. The expression levels of (b) ADAM9, (c) HSP27, (d) HSP70, (e) PCNA, (f) Bax, (g) Bcl-2, (h) caspase-3, (i) VEGF, and (j) p-STAT3 quantified using Gel-Pro Analyzer 4.0 software (Media Cybernetics Inc.). Band intensities normalized to *β*-actin. AU = arbitrary unit. ^∗∗^*P* < 0.01 and ^∗^*P* < 0.05: significant differences between the normal+ADAM9-sgRNA3, saline+alcohol, ADAM9-sgRNA+alcohol, and normal group. ^##^*P* < 0.01 and ^#^*P* < 0.05: significant differences between the normal+ADAM9-sgRNA3, ADAM9-sgRNA+alcohol, and saline+alcohol groups. ^△△^*P* < 0.01 and ^△^*P* < 0.05: significant difference between the ADAM9-sgRNA+alcohol group and the normal+ADAM9-sgRNA3 group.

The article "Silencing the ADAM9 Gene through CRISPR/Cas9 Protects Mice from Alcohol-Induced Acute Liver Injury" was published in 2022. Journal: Biomed Res Int.

## Data Availability

If other people apply, data will be available for them.
